# Risk of Acute Respiratory Distress Syndrome in Community-Acquired Pneumonia Patients: Use of an Artificial Neural Network Model

**DOI:** 10.1155/2023/2631779

**Published:** 2023-02-07

**Authors:** Jipeng Mo, Shihui Ling, Mingxia Yang, Hui Qin

**Affiliations:** ^1^Department of Critical Care Medicine, The Affiliated Changzhou No. 2 People's Hospital of Nanjing Medical University, Changzhou 213003, Jiangsu, China; ^2^Department of Emergency, The Affiliated Changzhou No. 2 People's Hospital of Nanjing Medical University, Changzhou 213003, Jiangsu, China; ^3^Department of Respiratory and Critical Care Medicine, The Affiliated Changzhou No. 2 People's Hospital of Nanjing Medical University, Changzhou 213003, Jiangsu, China

## Abstract

This study aimed to explore the independent risk factors for community-acquired pneumonia (CAP) complicated with acute respiratory distress syndrome (ARDS) and to predict and evaluate the risk of ARDS in CAP patients based on artificial neural network models (ANNs). We retrospectively analyzed eligible 989 CAP patients (632 men and 357 women) who met the criteria from the comprehensive intensive care unit (ICU) and the respiratory and critical care medicine department of Changzhou Second People's Hospital, Jiangsu Provincial People's Hospital, Nanjing Military Region General Hospital, and Wuxi Fifth People's Hospital between February 2018 and February 2021. The best predictors to model the ANNs were selected from 51 variables measured within 24 h after admission. By using this model, patients were divided into a training group (*n* = 701) and a testing group (*n* = 288 patients). Results showed that in 989 CAP patients, 22 important variables were identified as risk factors. The sensitivity, specificity, and accuracy of the ANNs model training group were 88.9%, 90.1%, and 89.7%, respectively. When ANNs were used in the test group, their sensitivity, specificity, and accuracy were 85.0%, 87.3%, and 86.5%, respectively; when ANNs were used to predict ARDS, the area under the receiver operating characteristic (ROC) curve was 0.943 (95% confidence interval (0.918–0.968)). The nine most important independent variables affecting the ANNs models were lactate dehydrogenase (100%), activated partial thromboplastin time (84.6%), procalcitonin (83.8%), age (77.9%), maximum respiratory rate (76.0%), neutrophil (75.9%), source of admission (68.9%), concentration of total serum kalium (61.3%), and concentration of total serum bilirubin (50.4%) (all important >50%). The ANNs model and the logistic regression models were significantly different in predicting and evaluating ARDS in CAP patients. Thus, the ANNs model has a good predictive value in predicting and evaluating ARDS in CAP patients, and its performance is better than that of the logistic regression model in predicting the incidence of ARDS patients.

## 1. Introduction

Community-acquired pneumonia (CAP) is one of the most common infectious diseases in the world, and the nosocomial mortality of CAP patients is about 13% [1]. Studies have indicated that about 21% of patients will develop severe CAP and need treatment in the intensive care unit (ICU), 26% of patients in the ICU need mechanical ventilation, and 29% of CAP patients will develop acute respiratory distress syndrome (ARDS) [2]. The mortality in severe CAP patients with concurrent ARDS is up to 30%, which may be related to the poorly recognized pathophysiology of ARDS [3]. Furthermore, the mortality of patients with ARDS associated with CAP is independently associated with delayed admission to the ICU, an increase in medical costs, and a decrease in long-term quality of life [4].

Prediction of ARDS in CAP patients is mainly based on their clinical symptoms, degree of hypoxia (arterial blood gas analysis), lung imaging findings, and reliable biomarkers [5]. With the development of techniques used for the detection of biomarkers that can reflect the pathophysiological mechanism of diseases and the introduction of the US-European Consensus Standard [6], some feasible biomarkers have been identified to be used to predict the concurrent ARDS in CAP patients, such as plasma endocrine proteins [7], T lymphocytes [8], interleukin-8 [4], neutrophil traps [9], and angiogenesis-2 [10]. However, the use of biomarkers remains controversial. An artificial neural network (ANNs) model is a nonlinear mathematical model, and its unique working principle in the analysis of characteristics of data has almost no restrictions, which helps to fit complex multifactorial diseases with good sensitivity and specificity. Thus, ANNs have been used in the diagnosis and prognostic analysis of clinical diseases [11].

No risk prediction models have been proposed to predict the clinical ARDS in CAP patients. Therefore, it is particularly important to assess the risk of concurrent ARDS in CAP patients. In this retrospective study, a predictive model was constructed to predict the concurrent ARDS in CAP patients, which may provide information for the prevention of ARDS in CAP patients.

## 2. Materials and Methods

### 2.1. Ethics Statement

This retrospective case-control observational study was conducted according to the guidelines of the Declaration of Helsinki and was approved by the ethics committee of our hospital. This was a retrospective study that was approved by the institutional review board, but patient-specific informed consent was not obtained. This study was approved by the Ethics Committee of Changzhou Second People's Hospital, which is affiliated with Nanjing Medical University (IRB: 2020YLJSE086). Furthermore, all the data were provided only to investigators with privacy protection. All the raw data were collected according to the procedures outlined in the epidemiological guidelines.

### 2.2. Patients and Clinical Characteristics

There were 2,228 CAP patients (1,336 men and 892 women) randomly included from the comprehensive intensive care unit (ICU) and the respiratory and critical care medicine departments of Changzhou Second People's Hospital, Jiangsu Provincial People's Hospital, Nanjing Military Region General Hospital, and Wuxi Fifth People's Hospital between February 2018 and February 2021.

Diagnostic criteria for CAP in China [1] are as follows: (a) it was acquired in the community. (b) There were pneumonia-related clinical manifestations such as (1) recent aggravation of cough, sputum, or existing respiratory disease, with or without concentrated sputum/chest pain/dyspnea/hemoptysis; (2) fever; (3) pulmonary consolidation signs and (or) wet rales; (4) peripheral white blood cells >10 × 10^9^/L or <4 × 10^9^/L, with or without left nucleus migration. (c) Chest imaging revealed a newly patchy infiltrating shadow, leaf/segment solid contrast, ground-glass opacity, or interstitial changes with or without pleural effusion. A clinical diagnosis was established once it met one of the *a*, *c*, and *b* characteristics, when pulmonary tuberculosis, pulmonary tumors, noninfectious pulmonary interstitial disease, pulmonary edema, atelectasis, pulmonary embolism, pulmonary eosinophil infiltration, or pulmonary vasculitis were excluded. Berlin 2012 diagnostic criteria for adult ARDS [12]: (1) time: within 1 week of known clinical onset or aggravation; (2) thoracic imaging findings: double lung density, pleural effusion, lobe/lung collapse, or nodules not fully explained on X-ray or CT; (3) causes of pulmonary edema: respiratory failure not fully explained by heart failure or fluid overload; (4) oxygenation dysfunction: mild: 200 mmHg < PaO_2_/FIO_2_ ≤ 300 mmHg, and positive end-expiratory pressure (PEEP) = 5 cmH_2_O; moderate: 100 mmHg < PaO_2_/FIO_2_ ≤ 200 mmHg, and PEEP = 5 cmH_2_O; severe severity: PaO_2_/FIO_2_ ≤ 100 mmHg, and PEEP = 5 cmH_2_O. If the altitude was above 1,000 m, the correction factor should be calculated as PaO_2_/FIO_2_ = atmospheric pressure/760.

According to the 51 clinical risk factors of CAP patients with statistically significant were recorded as follows: age, gender, source of admission (emergency, outpatient), maximum temperature (MT), maximum heart rate (MHR), maximum systolic blood pressure (MSBP), maximum respiratory rate (MRR), urine volume within 24 h, complement C4 (C4), hypertension, diabetes, c-reactive protein (CRP), procalcitonin (PCT), erythrocyte sedimentation rate (ESR), white blood cell count (WBC), neutrophil count (NEUT), lymphocyte count (LYM), eosinophil count (EO), fibrinogen equivalent unit (FEU), fibrinogen (FBG), activated partial thromboplastin time (APTT), alkaline phosphatase (ALP), albumin (ALB), total protein (TP), total bilirubin (TBIL), prealbumin (PA), alanine aminotransferase (ALT), aspartate aminotransferase (AST), lactate dehydrogenase(LDH), creatine kinase isoenzyme (CK-MB), troponin I (TNI), B-type natriuretic peptide (BNP), creatinine (CREA), blood urea nitrogen (BUN), uric acid (UA), red blood cell count (RBC), hemoglobin (HGB), platelet (PLT), glucose (GLU), total serum kalium (K^+^) level, total serum natrium (Na^+^) level, total serum magnesium (Mg^2+^) level, fraction of inspiration O_2_ (FiO_2_), potential of hydrogen (pH), oxygen partial pressure (PaO_2_), partial pressure of carbon dioxide (PaCO_2_), lactic acid (LAC), glasgow coma scale (GCS) score, nutritional risk score, lung injury score, and acute physiology and chronic health evaluation (APACHE). In addition, the gender, age, and source of admission (emergency department and outpatient department), the patient had the worst examination result within 24 h of admission.

### 2.3. Inclusion and Exclusion Criteria

CAP patients: Inclusion criteria were as follows: the patients with the initial diagnosis of CAP within 24 h served as CAP patients, and CAP was diagnosed based on the criteria from the Respiratory Society of the Chinese Medical Association and the Guidelines for the Diagnosis and Treatment of Adult Community-Acquired Pneumonia in China (2020 edition). Exclusion criteria were as follows: (1) There was confirmed severe respiratory dysfunction before the onset of CAP, such as acute respiratory distress syndrome, acute respiratory failure, severe pulmonary edema, and acute exacerbation phase of chronic obstructive pulmonary disease; (2) patients were admitted to hospital for pneumonia more than 2 times or patients required long-term oxygen therapy after tracheostomy; (3) the patient was transferred from other departments to the general ICU or the Department of Respiratory and Critical Care Medicine during the hospitalization; (4) presence of hospital-acquired pneumonia during hospitalization; (5) cardiac pulmonary edema during hospitalization; (6) presence of other risk factors on admission, cancer, heart failure or kidney failure, blood disease, and tuberculosis; (7) the disease condition was stable or normal within 48 h after admission; (8) patients with >30% deletions in the clinical risk variables; (9) patients with missing data in the identified clinical variables; (10) hospital stay <24 h; (11) incomplete clinical information.

### 2.4. Artificial Neural Networks Model

The 3-layer network model, including an input layer, output layer, and hidden layer, is mainly used to analyze the data. The independent variable *Xi*(*i*=1,2,3 … *n*) is used as the input neurons; the dependent variable *Y*_*j*_ (*j* = 0, 1) is the output neurons, and the output layer is ARDS (no ARDS = 0; ARDS = 1); its transfer parameters are expressed by the activation function identity. ANNs were conducted based on the building block of the single implicit layer with the classes separated through the following equation:

(1) $$\begin{array}{c} y=w\_1*x\_1+w\_2*x\_2+\cdots +w\_i*x\_i+b, \end{array}$$

where *x* represents the input, *w*_*i* represents the weights, *b* represents the bias, and *y* represents the output.

With *K* as the number of hidden layers, all data are normalized by $\bar{x}=\left(X-X\;\min\right)/\left(X\;\max\;–X\;\min\right)$. By gradually increasing and decreasing the number of neurons in the hidden layer, the number of hidden layer neurons that give the network sufficient generalization and output accuracy is selected. Finally, *K* is determined as 1 hidden layer including five neuronal units. As synaptic weights, its transfer function is dominated by the hyperbolic tangent function and reported by the activation function tangent curve. All the data were divided into a training dataset and a validation dataset at 7 : 3 ratio. The training dataset is used for network learning to build the prediction model, and the validation dataset is used to evaluate the performance of the model.

### 2.5. Logistic Regression Model

The logistic regression (LR) model is a generalized linear regression model, similar to the ANN model. In this model, the dependent variables serve as the output one, which is a binary variable (“no ARDS = 0,” “ARDS = 1”). The independent variables are the clinical risk factors as initial input ones, such as age, sex, heart rate, and hypertension. Independent variables can be continuous or categorical variables. In the logistic regression analysis, the weight of each independent variable can be obtained, and the risk factors for developing ARDS are determined. Meanwhile, the weight can be used to predict the likelihood of developing ARDS in a specific person based on the risk factors. The combination of each predictor was employed to predict the ARDS by a link function, logistic. The dataset was randomly divided into training and validation groups at a 1 : 1 ratio and the dataset in the training group was used to construct the LR model.

### 2.6. Statistical Analysis

All data were analyzed using SPSS version 26.0 statistical software. Data with normal distribution are expressed as mean ± standard deviation (*X* ± SD), and compared with an independent sample *t*-test between two groups. Data without normal distribution are expressed as medians (P25–P75), and compared with a nonparametric Kruskal–Wallis rank-sum test between the groups. Categorial data are expressed by frequency and rate, and compared between groups by the chi-square test. A value of *P* < 0.05 was considered statistically significant. ANN analysis was performed using SPSS Clementine11.1. The LR and ANN models were established to predict the risk of developing ARDS in CAP patients. Predictive performance was evaluated by sensitivity (SEN) and specificity (SPE). Dichotomous variables were created from continuous variables according to clinically important cut-off values. (MathWorks Institute, USA) was used to delineate the receiver operating characteristic (ROC) curves, and the area under the ROC curve (AUC) was calculated.

## 3. Results

### 3.1. Patients' Characteristics

A total of 2228 patients who were admitted due to the initial diagnosis of CAP were included in this study. There were 989 patients (632 men and 357 women) with a mean age of 68.48 ± 29.49 years were diagnosed with CAP alone, and 323 (32.7%) CAP patients developed ARDS (Figure 1). According to the exclusion criteria of clinical risk variables (1) the missing observed value of risk variables is >15%; (2) retain the most representative risk variables representing the same functional index; (3) the risk variable data is seriously skewed in distribution; (4) exclude the risk variables of blood gas analysis, and affect the accurate value of arterial blood gas analysis when using the ventilator. Finally, 25 clinical risk factors were collected for each patient such as gender, age, MHR, MT, MSBP, MRR, source of admission (emergency, outpatient), hypertension, diabetes, CRP, PCT, ESR, NEUT, EO, FEU, APTT, TBIL, ALB, LDH, CREA, HGB, PLT, GLU, K^+^, and Na^+^. Results of univariate analysis are shown in Table 1, and a *P* < 0.05 indicates the significant differences between the ARDS groups compared with the non-ARDS groups.

### 3.2. Prediction of ARDS with ANN Model

According to the ANN analysis, the input layer was the risk factor, and the 22 risk factors were entered successively according to the numbers *X*_1_–*X*_19_, including the dependent variables *X*_1_–*X*_4_, gender *X*_1_, admission source *X*_2_, hypertension *X*_3_, and diabetes *X*_4_. Covariates *X*_1_–*X*_19_ were entered sequentially, including age *X*_1_, heart rate *X*_2_, MRR *X*_3_, CRP *X*_4_, PCT *X*_5_, ESR *X*_6_, NEUT *X*_7_, EO *X*_8_, FEU *X*_9_, APTT *X*_10_, TBIL *X*_11_, ALB *X*_12_, LDH *X*_13_, CREA *X*_14_, HGB *X*_15_, GLU *X*_16_, PLT *X*_17_, K^+^*X*_18_, and Na ^+^ *X*_19_. The output layer was ARDS (no ARDS = 0, ARDS = 1). The number of hidden layers as interneurons was set as 5. The topological stratification structure of the neural network model is plotted (Figure 2).

The BP neural network model was built using the training dataset. The sensitivity, specificity, and accuracy of the ANN model were 88.9%, 90.1%, and 89.7%, respectively, in the training group. This indicates that the ANN model has good recognition ability. In the test group, the sensitivity, specificity, and accuracy of the ANN model were 85.0%, 87.3%, and 86.5%, respectively (Table 2). When the ANN model was used to predict ARDS, the AUC was 0.943, and the 95% confidence interval (CI) was 0.926–0.928 (Figure 3). In the training group and the ANNs model in the test group, the error rates of prediction were 10.3% and 13.5%, respectively, indicating that the two datasets have good accuracy in the prediction model. In our study, the fit of ARDS and non-ARDS predictions were compared with the Hosmer and Lemeshow test, and results showed that ARDS fits were better than those of non-ARDS, indicating that the ANN model is more suitable for predicting the occurrence of ARDS.

The importance of each predictor of the BP neural network was determined when the normalized importance analysis was performed. Among the 23 independent variables of ARDS, LDH, APTT, PCT, age, MRR, NEUT, source of admission, K^+^, and TBIL were the nine most important ones. After standardization, the nine independent variables were LDH (100%), APTT (84.6%), PCT (83.8%), age (77.9%), MRR (76.0%), NEUT (75.9%), admission source (68.9%), K^+^(61.3%), and TBIL (50.4%) (all >50%) (Figure 4).

### 3.3. Prediction of ARDS with LR Model

Univariate LR analysis identified 25 variables related to ARDS. Among these factors, 22 variables were significantly different between ARDS patients and non-ARDS patients (*P* < 0.05). Age, gender, MHR, MRR, admission source (emergency, outpatient), hypertension, CRP, PCT, ESR, NEUT, EO, FEU, APTT, TBIL, ALB, LDH, CREA, HGB, PLT, GLU, K^+^, and Na^+^ were included into the multivariate LR analysis as predictive variables. The final LR equation was logit (*P*) = −2.745 + 3.948 × admission source + 0.004 × CRP + 0.045 × PCT + 0.008 × ESR − 0.009 × NEUT − 0.47 × ALB + 0.03 × LDH, and *P* represents the predicting probability of the LR model (Table 3). When it was used in the validation dataset, the LR model had an SEN of 89.2%, an SPE of 88.1%, and an accuracy of 88.5% (Table 2).

### 3.4. Comparison of ANN Model with LR Model

The evaluation metrics of BP-ANNs and LR models were compared. The results showed no significant differences in the SEN, SPE, accuracy, and AUC between them (*P* > 0.05). The AUC was calculated in the LR and ANN models established using the validation dataset and used to identify the ARDS. The AUC of the ANN model was 0.943 (95% CI: 0.918–0.968), and the AUC of the LR model was 0.942 (95% CI: 0.923–0.961) (Table 4).

## 4. Discussion

CAP developed severe CAP and needs intensive care patients, the most common complication is ARDS. ARDS is a heterogeneous syndrome, including direct and indirect causes of lung injury, and pulmonary ARDS is a CAP sepsis-like inflammatory reaction and alveolar endothelial injury [13]. Some studies have found that pulmonary edema in ARDS is unspecific, and may further increase the mortality of ARDS patients [14, 15]. Thus, the development of a model for the prediction of ARDS in CAP patients may be helpful for the early monitoring and management of severe diseases and the reduction of risk for ARDS in CAP patients.

This study for the first time investigates the predictive model of ARDS in CAP patients with conventional variables. In this model, all objective and commonly used clinical variables collected within 24 h after admission were included. The predictive model of ARDS in CAP patients constructed with the ANN model has good predictive and calibration power. In our study, LDH, APTT, PCT, age, MRR, NEUT, admission source, K^+^, and TBIL played important roles in predicting the occurrence of ARDS in CAP patients, and some previous studies have investigated the specific risk factors of ARDS in CAP patients. As a key enzyme in the glycolytic pathway, LDH is a cytoplasmic enzyme in most organs, which is associated with an inflammatory response and cellular damage. Zhou et al. found that bacterial or viral mRNA clearance is highly correlated with LDH level, and CAP patients infected by bacteria or viruses may have inflammasome activation, induction of apoptosis, and invasive symptoms, which can partly explain the association of LDH with CAP and ARDS [16]. Zhou et al. also found that an elevated LDH level in admitted patients was strongly associated with the risk of developing ARDS [16]. Pathophysiologically, ARDS is mainly characterized by inflammatory cell migration, fiber proliferation, and apoptosis, the imbalance between hypercoagulability and inflammation may lead to excessive inflammation and accelerate the fibrin deposition in the alveoli [17]. CAP patients develop severe pneumonia, in which neutrophils gradually form external neutrophil traps, further increasing lung endothelial and epithelial cell damage, which leads to the occurrence of ARDS and acute respiratory failure. Immune thrombosis is a key manifestation of ARDS. Grasselli et al. found that the fibrin-rich exudates due to coagulation activation and inhibition were the core event in the pathophysiology of ARDS [18], and the coagulation function (fibrinolysis) was related to the development of ARDS. Studies have confirmed that ARDS patients have severe coagulation dysfunction, and the liver peak test has demonstrated a strong association of TBIL with ARDS in patients receiving mechanical ventilation in the ICU [19]. It has been shown that pneumonia is unlikely to be responsible for the elevation of procalcitonin. However, the elevated PCT may be related to the longer duration of mechanical ventilation in patients with severe pneumonia in the ICU [20]. Tang et al. found that procalcitonin was related to the acute exacerbation of inflammation and could be used to assess the severity of CAP as a risk factor for ARDS [21]. The immunity may gradually compromise with age, easily leading to bacterial and viral invasion [22], which is also confirmed by the significantly older age of CAP patients with ARDS in this study as compared to those without ARDS. Pensier et al. employed protective ventilation to improve lung tension, which is conducive to the further improvement of ARDS [23]. The source of admission is also a risk factor for ARDS in CAP patients, and the incidence of ARDS is significantly higher in patients admitted to the emergency department than in those of other sources [24]. In patients with CAP secondary to sepsis or ARDS, impaired hypoxic pulmonary vasoconstriction (HPV) may lead to fluid perfusion mismatching and hypoxia. The voltage-gated potassium channels have been shown to be one of the key regulators of HPV. ATP-sensitive potassium channels increase in case of endotoxemia and are also involved in the pathogenesis of alveolar epithelial barrier failure, explaining the importance of potassium in the ARDS [25, 26]. Fu et al. reported that high body temperature, high systolic blood pressure, and diabetes were not associated with the development of ARDS [27]. Our results were consistent with those reported in available studies. In addition, some studies have mentioned that low levels of albumin, hemoglobin, and fibrinogen are risk predictors of ARDS [28]. These metrics were also used as potential predictors, and new predictors were added to the aforementioned factors. Furthermore, the study by Dzierba et al. concluded that platelet count decreased and ARDS occurred in patients with septic shock, and they were unrelated to the occurrence of ARDS in the nonseptic shock subgroup [29], which was inconsistent with our findings. The role of platelets in the pathogenesis of ARDS may be probably mediated by platelet-related inflammatory responses and disseminated intravascular coagulation. Thrombocytopenia is a key feature of the systemic inflammatory response [30, 31], which was confirmed in all ARDS patients as compared to non-ARDS patients in this study.

CAP patients have a high risk for ARDS. In the present study, a predictive model was established to predict ARDS in CAP patients. The previous pre-established ARDS model based on different risk factors on admission has a good predictive ability and focuses on the prediction of ARDS in CAP patients. The clinical outcomes and biomarker characteristics of CAP patients with ARDS differ from patients with ARDS unrelated to non-CAP risk factors, which reflects the unique potential clinical factors and the special pathogenic mechanism of CAP [22]. In the present study, the BP-ANNs model was compared with the LR model, and results showed the two models were compared in the SEN, SPE, accuracy, and AUC (*P* > 0.05). ANN was used in this study. Compared with the traditional LR, ANN is a nonlinear mathematical model, and its unique working principle has almost no restrictions on the characteristics of data used for analysis, which helps fit complex multifactorial diseases and has good sensitivity and specificity [11]. Therefore, ANN was employed to construct a model for the prediction of ARDS in CAP patients, and results showed its AUC was 0.943, showing a good predictive performance. Based on the ANN method, the predictive power reached 89.7% in the trained dataset and 86.5% in the verified dataset. The decrease in predictive power in the trained dataset may be related to the small sample size. In this study, the number of predictors for the proportion of ARDS was limited, aiming to avoid this bias. Although this only slightly affected the predictive power of the model, it had a large impact on the model calibration. Overall, the predictive model of this study systematically overestimated the risk of developing ARDS due to the relatively small sample size in the cohort.

There were still limitations in this study: First, the sample size was small in patients with ARDS, and thus more clinical studies with a large sample size are needed to improve the accuracy of the prediction model and confirm our study. Second, some predictors have been repeatedly mentioned in the studies, such as smoking, body mass index, acute physiology, and chronic health evaluation II, complement C3, but they were not included as potential predictors in this study. Third, there was an overlap between some predictors in this study (FEU, APTT). However, the aim of this study was not to establish an independent association between risk factors and ARDS. Instead, our study aimed to determine the combination of variables that can achieve the best predictive performance for CAP-related ARDS. Fourth, the case size in the present study was not very well established, due to the heterogeneity in the ARDS heterogenicity, compromising the identification ability of these predictors. Fifth, early lack of CAP patients with a conclusion urea respiratory rate and age 65 (CURB-65) for grouping, To further predict the high-risk group (CURB-65 score 3 points) model. Sixth, causal inference is an important aspect of machine learning [32], but the current predictors in this study are not necessarily causal factors for ARDS. Therefore, more prospective multicenter randomized controlled studies with a large sample size are warranted to confirm our findings in the future.

## 5. Conclusions

In conclusion, the predictive model constructed in this study based on the ANN model using the indicators collected early after admission can be used to calculate and stratify ARDS in CAP patients. Specifically, the model can be used to calculate risk and intervene in the early targeting of meaningful markers in this study. The model may provide a reference for the early allocation of medical resources and help to guide the clinical management of CAP patients.

## Figures and Tables

**Figure 1:** CAP patients enrollment according to the inclusion and exclusion criteria. *Note*. CAP, community-acquired pneumonia.

**Figure 2:** Topological stratification structure of the ARDS prediction model in CAP patients based on an artificial neural network model. *Note.* CAP, community-acquired pneumonia; ARDS, acute respiratory distress syndrome.

**Figure 3:** ROC curve of the ARDS prediction model in CAP patients based on an artificial neural network model. *Note.* CAP, community-acquired pneumonia; ARDS, acute respiratory distress syndrome; AUC, the area under the ROC curve.

**Figure 4:** Normalized importance distribution of the influence of input layer independent variables on the output layer in a concurrent ARDS prediction model for CAP patients based on an artificial neural network model. *Note.* CAP, community-acquired pneumonia; ARDS, acute respiratory distress syndrome.

**Table 1:** Univariate analysis of factors related to ARDS in CAP patients.

Variable	Statistical method	Non-ARDS group (IQR) (*n* = 666)	ARDS group (IQR) (*n* = 323)	*χ* ^2^/*t* value	*P* value
Demographic characteristics					
Age (years)	Rank-sum test	68.0 (55.0–78.0)	73.2 (67.0–83.0)	7.260	<0.001
Gender (%)	Chi-square test			18.650	<0.001
Man		395 (59.3%)	237 (73.4%)		
Woman		271 (40.7%)	86 (26.6%)		
Clinical characteristics					
Hypertension (%)	Chi-square test	297 (44.6%)	181 (56.0%)	11.400	≤0.001
Diabetes (%)	Chi-square test	146 (21.9%)	87 (26.9%)	0.100	0.825
MSPB (mmHg)	Rank-sum test	126.0 (114.0–138.0)	124.0 (107.0–139.0)	−1.740	0.081
MT (°C)	Rank-sum test	36.8 (36.5–37.3)	37.0 (36.5–37.6)	1.890	0.058
MRR (sub/min)	Rank-sum test	18.0 (18.0–20.0)	22.0 (19.0–29.0)	11.200	<0.001
MHR (sub/min)	Rank-sum test	85.0 (76.0–94.0)	97.0 (82.0–112.0)	4.300	<0.001
Source of admission	Chi-square test			567.940	<0.001
Outpatient (%)		82 (12.3%)	293 (90.7%)		
Emergency (%)		584 (87.7%)	73 (89.0%)		
Laboratory findings					
CRP (mg/L)	Rank-sum test	28.0 (6.6–81.3)	85.3 (28.9–134.1)	9.190	<0.001
PCT (ng/mL)	Rank-sum test	0.1 (0–0.3)	0.8 (0.2–6.5)	15.940	<0.001
ESR (mm/h)	Rank-sum test	30.0 (15.0–58.0)	50.0 (25.0–77.0)	6.660	<0.001
NEUT (×109/L)	Rank-sum test	5.0 (3.3–7.6)	10.2 (6.6–13.9)	12.930	<0.001
EO (×10^9/L)	Rank-sum test	0.1 (0–0.2)	0 (0–0.2)	−5.970	<0.001
FEU (mg/l)	Rank-sum test	0.7 (0.3–1.6)	2.7 (1.4–6.4)	15.580	<0.001
APTT (sec)	Rank-sum test	28.9 (27.0–31.8)	32.1 (28.8–36.0)	8.510	<0.001
TBIL (umol/L)	Rank-sum test	9.1 (6.6–13.0)	13.7 (9.0–20.2)	9.120	<0.001
ALB (g/L)	Rank-sum test	37.0 (32.5–40.9)	31.0 (27.4–35.4)	13.170	<0.001
LDH (U/L)	Rank-sum test	195.0 (164.0–235.0)	288.5 (204.0–436.0)	12.440	<0.001
CREA (*μ*mol/L)	Rank-sum test	64.1 (52.3–80.0)	80.1 (55.3–130.0)	6.680	<0.001
HGB (g/L)	Rank-sum test	125.0 (110.0–138.0)	110.2 (92.0–129.0)	−7.200	<0.001
PLT (×109)	Rank-sum test	214.0 (167.0–267.0)	197.0 (125.0–257.0)	−3.480	0.001
GLU (mmol/L)	Rank-sum test	5.6 (4.9–7.5)	8.2 (6.5–11.0)	11.350	<0.001
K^+^	Rank-sum test	3.9 (3.6–4.2)	4.0 (3.5–4.4)	3.340	0.001
Na^+^	Rank-sum test	138.8 (136.1–141.0)	137.0 (132.8–142.5)	−2.57	0.010

*Note.* IQR, interquartile ranges; ARDS, acute respiratory distress syndrome; CAP, community-acquired pneumonia; MSPB, maximum systolic blood pressure; MT, maximum temperature; MRR, maximum respiratory rate; MHR, maximum heart rate; CRP, c-reactive protein; PCT, procalcitonin; ESR, erythrocyte sedimentation rate; NEUT, neutrophil count; EO, eosinophil count; FEU, fibrinogen equivalent unit; APTT, activated partial thromboplastin time; TBIL, total bilirubin; ALB, albumin; LDH, lactate dehydrogenase; CREA, creatinine; HGB, hemoglobin; PLT, platelet; GLU, glucose; K^+^, the concentration of total level of serum kalium; Na^+^, the concentration of total level of serum natrium.

**Table 2:** Accuracy of ARDS prediction in CAP patients based on training and testing datasets from ANNs.

Group	Actual measurement	Total	Calculate		
			Non-ARDS	ARDS	Accuracy rate (%)
Training	Non-ARDS	485	437	48	90.1 (437/485)
	ARDS	216	24	192	88.9 (192/216)
	Total	701	461	240	89.7 (629/701)

Testing	Non-ARDS	181	158	23	87.3 (158/181)
	ARDS	107	16	91	85.0 (91/107)
	Total	288	174	114	86.5 (249/288)

*Note.* ARDS, acute respiratory distress syndrome; CAP, community-acquired pneumonia; ANNs, artificial neural network models.

**Table 3:** Multivariate analysis of factors related to ARDS in CAP patients.

Variables	*B*	S.E	Wald	Sig	Exp (*B*)	95% CI for exp (*B*)
Source of admission	3.948	0.246	258.222	≤0.001	51.822	32.018–83.875
CRP	0.004	0.002	5.083	0.024	1.004	1.000–1.007
PCT	0.045	0.012	14.705	≤0.001	1.046	1.022–1.070
ESR	0.008	0.003	4.666	0.031	1.008	1.001–1.014
NEUT	−0.009	0.003	11.853	0.001	0.991	0.986–0.996
ALB	−0.047	0.019	6.144	0.013	0.954	0.920–0.990
LDH	0.003	0.001	21.621	≤0.001	1.003	1.002–1.004
Constant	−0.2743	0.782	12.292	≤0.001	0.064	

*Note.* ARDS, acute respiratory distress syndrome; CAP, community-acquired pneumonia; CRP, c-reactive protein; PCT, procalcitonin; ESR, erythrocyte sedimentation rate; NEUT, neutrophil count; EO, eosinophil count; ALB, albumin; and LDH, lactate dehydrogenase.

**Table 4:** Comparison of the ANNs model and LR model in predicting ARDS secondary to CAP in the test dataset.

Variable	ANNs model	LR model	Difference between models (95% CI)	*P* value
Sensitivity	85.0%	89.2%	4.2% (1.2–6.9%)	0.093
Specificity	87.3%	88.1%	0.8% (0.4–1.4%)	0.405
Accuracy	86.5%	88.5%	2.0% (1.1–3.4%)	0.136
AUC	0.943 ± 0.025	0.942 ± 0.019	0.001 (0.000–0.002)	0.180

*Note.* ANNs, artificial neural networks; LR, logistic regression; ARDS, acute respiratory distress syndrome; CAP, community-acquired pneumonia; AUC, the area under ROC (receiver operating characteristic) curve.

## Data Availability

The data used to support the findings of this study are available from the corresponding author upon request.
